The article "Long non‐coding RNA PGM5‐AS1 promotes epithelial‐mesenchymal transition, invasion and metastasis of osteosarcoma cells by impairing miR‐140‐5p‐mediated FBN1 inhibition" was retracted in 2023. Reasons: duplicated images; original data or images not available; unreliable results or conclusions.

# Long non‐coding RNA PGM5‐AS1 promotes epithelial‐mesenchymal transition, invasion and metastasis of osteosarcoma cells by impairing miR‐140‐5p‐mediated FBN1 inhibition

**DOI:** 10.1002/1878-0261.12711

**Published:** 2020-08-19

**Authors:** Wei Liu, Pengcheng Liu, Hang Gao, Xu Wang, Ming Yan

**Affiliations:** ^1^ Department of Spine Surgery The First Hospital of Jilin University Changchun China; ^2^ Department of Hand and Foot Surgery The First Hospital of Jilin University Changchun China; ^3^ Department of Bone and Joint Surgery The First Hospital of Jilin University Changchun China; ^4^ Department of Colorectal and Anal Surgery The First Hospital of Jilin University Changchun China

**Keywords:** fibrillin‐1, long noncoding RNA PGM5‐AS1, microRNA‐140‐5p, osteosarcoma

## Abstract

Osteosarcoma is an uncommon tumor occurring in bone, accompanied by elevated incidence and reduced rate of healing. Epithelial‐to‐mesenchymal transition (EMT) serves as a conceptual paradigm to explain the invasion and metastasis of osteosarcoma and other cancers. Hence, developing effective therapeutic strategy to treat the EMT of osteosarcoma is essential. Here, we identified the molecular mechanism of long noncoding RNA (lncRNA) PGM5‐AS1 in EMT and progression of osteosarcoma. Microarray‐based analysis was employed to screen the osteosarcoma‐related differentially expressed lncRNAs. The levels of PGM5‐AS1 as well as microRNA‐140‐5p (miR‐140‐5p) and fibrillin‐1 (FBN1) in osteosarcoma tissues and cells were determined. Dual‐luciferase reporter gene assay, RNA pull‐down assay, and RNA immunoprecipitation assay were conducted to validate the relationship among PGM5‐AS1, miR‐140‐5p, and FBN1. Expression of PGM5‐AS1, miR‐140‐5p, and FBN1 was altered by overexpression, shRNA, mimic, or inhibitors in order to investigate how they regulated migration, invasion, and EMT of osteosarcoma cells *in vitro*. Loss‐ and gain‐of‐function approaches were employed in nude mice to detect their roles in tumorigenesis *in vivo*. Osteosarcoma tissues and cells exhibited low expression of miR‐140‐5p, but high expression of PGM5‐AS1 and FBN1. PGM5‐AS1 competitively bound to miR‐140‐5p to upregulate FBN1. Furthermore, hindering PGM5‐AS1 and FBN1 or overexpressing miR‐140‐5p dampened migration, invasion, and EMT of osteosarcoma cells *in vitro*. Furthermore, silencing PGM5‐AS1 or FBN1, or overexpressing miR‐140‐5p markedly inhibited tumorigenesis in nude mice *in vivo*. Taken together, PGM5‐AS1 depletion causes FBN1 reduction to retard osteosarcoma processes by negatively modulating miR‐140‐5p.

## Graphical abstract

In this study, we analyzed the modulatory role of PGM5‐AS1 in the progression and EMT of osteosarcoma. In osteosarcoma tissues and cells, PGM5‐AS1 and FBN1 are highly expressed, while miR‐140‐5p exhibits low expression. We reveal that PGM5‐AS1 specifically binds to miR‐140‐5p to silence the expression of FBN1, and thereby attenuate EMT, invasion, and migration of osteosarcoma *in vitro* as well as tumorigenesis *in vivo*. In this study, we analyzed the modulatory role of PGM5‐AS1 in the progression and EMT of osteosarcoma. In osteosarcoma tissues and cells, PGM5‐AS1 and FBN1 are highly expressed, while miR‐140‐5p exhibits low expression. We reveal that PGM5‐AS1 specifically binds to miR‐140‐5p to silence the expression of FBN1, and thereby attenuate EMT, invasion, and migration of osteosarcoma *in vitro* as well as tumorigenesis *in vivo*.

**Abbreviations**
ANOVA: analysis of variance
DMEM: Dulbecco's modified Eagle's medium
EMT: epithelial–mesenchymal transition
FBN1: fibrillin‐1
FISH: fluorescence *in* *situ* hybridization
GAPDH: glyceraldehyde‐3‐phosphate dehydrogenase
GEO: Gene Expression Omnibus
lncRNA: long noncoding RNA
miR‐140‐5p: microRNA‐140‐5p
miRNAs: microRNAs
MUT: mutant type
NC: negative control
oe: overexpression
RIP: RNA immunoprecipitation
sh: short hairpin
WT: wild‐type

## 1 Introduction

As a rare malignant bone tumor of mesenchymal origin, osteosarcoma presents with osteoblastic differentiation and malignant osteoid formation, accompanied by local swelling and pain (Yang and Wang, 2016). It is a neoplasm with high incidence in children and adults, but its highest incidence rate is among people aged > 65 years (Lindsey *et al*., 2017). The current treatment options include amputation, intricate limb‐sparing surgeries, and multiagent chemotherapy (Isakoff *et al*., 2015). However, the biology of osteosarcoma remains poorly understood. In spite of the current progress in osteosarcoma treatment, patients still diagnosed with metastasis and relapse accompanied by low survival rate (Luetke *et al*., 2014). Moreover, as a conceptual paradigm, epithelial–mesenchymal transition (EMT) explains the invasion of cancer cells during progression of cancers including osteosarcoma (Lv *et al*., 2016). Therefore, developing novel ways to deal with the EMT of osteosarcoma is in significant importance to inhibit the progression of osteosarcoma.

Long noncoding RNAs (lncRNAs), small transcripts that do not encode proteins, are involved in a variety of processes of diseases, including osteosarcoma (Yang *et al*., 2016). The expression of taurine‐upregulated gene 1 was high in osteosarcoma tissues, and blocking its expression attenuated the proliferation of osteosarcoma cells (Zhang *et al*., 2013). PGM5 is a phosphotransferase enzyme that catalyzes the conversion between glucose‐1‐phosphate and glucose‐6‐phosphate (Zhu *et al*., 2017a, 2017b,2017a, 2017b). PGM5‐AS1 is a lncRNA with high expression in anaplastic glioma (Wang *et al*., 2018a, 2018b,2018a, 2018b), suggesting that PGM5‐AS1 may be involved in the progression of tumors. In the present study, PGM5‐AS1 was identified to bind to miR‐140‐5p. MicroRNAs (miRNAs), which are small noncoding RNAs with a length of about 18–25 nucleotides, are also associated with diverse processes of tumors including osteosarcoma (Kobayashi *et al*., 2014). miR‐140‐5p was reported to participate in the survival and chemoresistance of osteosarcoma. Specifically, elevated expression of miR‐140‐5p increased autophagy and suppressed the cell proliferation induced by anticancer drugs (Meng *et al*., 2017; Wei *et al*., 2016). Moreover, we also determined in this study that miR‐140‐5p could directly target fibrillin‐1 (FBN1), which is a common extracellular matrix molecule involved in sequestering of growth factors (Sengle *et al*., 2012). Osteosarcoma cells with elevated FBN1 level were linked to system of bone and skeletal (Han *et al*., 2014). Thus, we postulated from previous results that PGM5‐AS1, miR‐140‐5p, and FBN1 may constitute an axis influencing the progression of osteosarcoma cell processes, and undertook a range of assays *in vitro* and *in vivo* to explore this pathway.

## 2 Materials and methods

### 2.1 Ethics statement

All procedures strictly conformed to the Ethics Committee and Experimental Animal Ethics Committee of the First, Second and Third Affiliated Hospitals of Jilin University and guided by the intentions of the *Declaration of Helsinki*. Ethical agreements were acquired from all participants by written informed consent prior to their inclusion in the study. The animal experiments were performed in strict accordance with the guiding principle of minimizing discomfort of the experimental animals.

### 2.2 Microarray‐based analysis

The Gene Expression Omnibus (GEO) database was applied to retrieve the microarray dataset related to osteosarcoma. Through ‘limma’ package, differentially expressed genes were retrieved with the threshold of |logFC| > 2 and *P‐*value* < *0.05. The location of PGM5‐AS1 expression was predicted, and the downstream miRNA target of PGM5‐AS1 was predicted using the lncATLAS database (http://lncatlas.crg.eu/) and the RAID database (https://www.baidu.com/baidu?&ie=utf‐8&word=ncbi%20geo), respectively. The TargetScan database (http://www.targetscan.org/vert_71/), mirDIP database (http://ophid.utoronto.ca/mirDIP/index.jsp#r), miRDB database (http://mirdb.org/miRDB/index.html), and miRmap database (https://mirmap.ezlab.org/) were adopted to predict the downstream target gene of miR‐140‐5p.

### 2.3 Tissue specimen samples

Osteosarcoma tissues were harvested from 73 patients with detailed clinical data who were pathologically diagnosed as osteosarcoma and received surgical resection in the First, Second and Third Affiliated Hospitals of Jilin University from January 2013 to December 2017. The patients (41 males and 32 females) had not received chemoradiotherapy prior to the surgery aged from 9 to 53 years with an average age of 26.68 ± 13.50. Among these patients, 33 patients were aged ≤ 20 years old and 40 patients were aged > 20 years old; 38 patients' tumor diameter was ≤ 5 cm, while 35 patients' tumor diameter was > 5 cm. Besides, adjacent normal bone tissues located 4 cm away from the osteosarcoma tissues were also collected from these patients. Osteosarcoma and adjacent normal bone tissues were evaluated by pathologists according to the standards set by the World Health Organization (Hu *et al*., 2014; Yuan *et al*., 2017).

### 2.4 Follow‐up

Follow‐up of the patients via phone or return visit continued until December 2018 with the observation of overall survival rate of these patients. The 66 cases (90.41%) had follow‐up of duration 5–36 months, with seven patients lost to follow‐up.

### 2.5 RNA *in situ* hybridization

The 463‐bp DNA fragment (corresponding to nucleotide position 142–585 bp of PGM5‐AS1) was cloned into the pSPT19 vector (10999644001; Sigma, Shanghai, China), and synthesis of antisense RNA probe was performed using the DIG RNA Labeling Kit (SP6/T7; 11175025910, Sigma). The DNA fragment sequence of PGM5‐AS1‐ISH was as follows: F, GATCGGAATTCCGGGTAAGAGAATGTCCGAAAG; R, GATGCAAGCTTCACCATGCTGTGCTGTAGAT. The double DIG‐labeled LNA microRNA probe (QIAGEN, Shanghai, China) for miR‐140‐5p was incubated with the paraffin‐embedded osteosarcoma tissue sections. Briefly, after being deparaffinized, the tissue sections were treated with proteinase K (Roche, Basel, Switzerland), hybridized with 300 ng·mL^−1^ probe at 60 °C for 16 h, then incubated with anti‐digoxigenin‐AP (AP‐conjugated Fab fragments) (11093274910; Roche) at 25 °C for 1 h, and finally added with BM Purple (11442074001; Roche) for color reaction. The cells with brown or brownish‐yellow‐stained nuclei were regarded as positive, and the positive expression rate was calculated as the number of positive cells divided by the total number of cells. The percentage of positive tumor cells was scored as follows: 0 (0%), 1 (1–10%), 2 (11–50%), and 3 (> 50%). The staining intensity was also clarified into four grades: 0 (negative), 1 (weak), 2 (moderate), and 3 (strong). The average value was obtained after random selection of five views. Scores were determined independently by two experienced pathologists (Fang *et al*., 2017; Sun and Qin, 2018; Taniue *et al*., 2016).

### 2.6 Cell culture and treatment

A normal cell line hFOB 1.19 [CBP60724; Culture Medium: Dulbecco's modified Eagle's medium (DMEM): F12 + 0.3 mg·mL^−1^ G418 + 10% FBS) was cultured with 5% CO_2_ at 34 °C as described previously (Bozycki *et al*., 2018) and five cell lines related to osteosarcoma: U2OS (CBP60238; Culture Medium: McCoy's 5a + 10% FBS), SaOS‐2 (CBP60742; Culture Medium: McCoy's 5a + 15% FBS), MG63 (CBP60233; Culture Medium: MEM + 10% FBS), HOS (CBP60787; Culture Medium: RPMI‐1640 Medium + 10% FBS), and SJSA1 (CBP60236; Culture Medium: RPMI‐1640 + 10% FBS), which were purchased from Cobioer Biotechnology Co., Ltd. (Nanjing, China) and cultured with 5% CO_2_ at 37 °C. The medium was renewed every day.

Osteosarcoma cells were plated into 6‐well plates (3 × 10^5^ cells/well). Upon attaining 50% cell confluence, short hairpin RNA (sh)‐negative control (NC), sh‐PGM5‐AS1‐1, sh‐PGM5‐AS1‐2, overexpression (oe)‐NC, oe‐PGM5‐AS1, inhibitor NC, miR‐140‐5p inhibitor, mimic NC, miR‐140‐5p mimic, or sh‐FBN1 was delivered into the cells following the procedures in the Lipofectamine 2000 kit (11668‐019; Invitrogen, Carlsbad, CA, USA). The mimic NC, miR‐140‐5p mimic, inhibitor NC, and miR‐140‐5p inhibitor, and plasmids were purchased from Shanghai GenePharma Co., Ltd. (Shanghai, China). Table 1 displays the sequences of shRNAs.

**Table 1:** shRNA sequences.

Item	Sequence	Company
sh‐PGM5‐AS1‐1	GGGTAAGAGAATGTCCGAAAG	Thermo Fisher
sh‐PGM5‐AS1‐2	GGTAAGAGAATGTCCGAAAGA	Thermo Fisher
sh‐FBN1	GCATGCACTTACGGATTTACT	Thermo Fisher

### 2.7 Reverse transcription–quantitative polymerase chain reaction

Total RNA extraction from samples was performed using TRIzol kit (16096020; Thermo Fisher Scientific, Sunnyvale, CA, USA). Five‐microgram portions of RNA were reversely transcribed into cDNA following procedures specified in the cDNA kit (K1622; Fermentas Inc., Ontario, CA, USA). The TaqMan MicroRNA Assay and TaqMan^®^ Universal PCR Master Mix were applied for reverse transcription–quantitative polymerase chain reaction (RT‐qPCR), which followed the guidelines of the TaqMan Gene Expression Assay Kit (Applied Biosystems, Foster City, CA, USA) (Xie *et al*., 2019). Table 2 shows the sequences of primers. The $2^{-\Delta \Delta C_{t}}$ method was employed to calculate the relative expression of the target genes that was standardized by U6 (miR‐140‐5p) and glyceraldehyde‐3‐phosphate dehydrogenase (GAPDH) (PGM5‐AS1 and FBN1).

**Table 2:** Primer sequences used in reverse transcription–quantitative polymerase chain reaction.

Gene	Primer sequence (5′–3′)
PGM5‐AS1	F: CGCAGAGTCGGAGAAGAGTC
	R: CGGACAGGCTGAAAGTACCA
FBN1	F: GGGTCAAAGATCACGTGCACAG
	R: TTGTCAAAGCAGACGGAGGTC
miR‐140‐5p	F: TGCGGCAGTGGTTTTACCCTATG
	R: CCAGTGCAGGGTCCGAGGT
U6	F: GCTTCGGCAGCACATATACTAAAAT
	R: CGCTTCACGAATTTGCGTGTCAT
GAPDH	F: ATGGAGAAGGCTGGGGCTC
	R: AAGTTGTCATGGATGACCTTG

### 2.8 Western blot assay

The bicinchoninic acid protein assay kit (Thermo Fisher Scientific) was adopted for total protein extraction, followed by measurement of protein concentration. Next, 30‐μg portions of total protein were separated by polyacrylamide gel electrophoresis and then electroblotted onto polyvinylidene fluoride membranes (Amersham Healthcare, Chicago, IL, USA). The membrane was then blocked by 5% nonfat milk at room temperature for 1 h, followed by overnight incubation at 4 °C in rabbit polyclonal antibodies (Abcam Inc., Cambridge, UK) against FBN1 (ab231094, 1 : 1000), E‐cadherin (ab15148, 1 : 500), N‐cadherin (ab76057, 1 : 1000), Vimentin (ab137321, 1 : 2000), and GAPDH (ab9485, 1 : 2500). The 1‐h membrane incubation was then conducted in secondary antibody to goat anti‐rabbit IgG H&L (ab6721, 1 : 3000; Abcam Inc.) tagged by horseradish peroxidase at room temperature for 1 h. Then, the membrane was scanned and developed using a chemiluminescence instrument (Gel Company, San Francisco, CA, USA). The analysis of relative protein expression was conducted using image‐pro plus 6.0 software (Media Cybernetics, Silver Spring, MD, USA).

### 2.9 Transwell assay

Cell migration was detected as follows: When in logarithmic growth phase, osteosarcoma cells were starved for 24 h until the final concentration of cells reached 2 × 10^5^ cells·mL^−1^. Subsequently, 0.2 mL of cell suspension and 700 μL of precooled DMEM encompassing 10% FBS were supplemented into the apical and basolateral chambers, respectively, followed by 24‐h culture at 37 °C with 5% CO_2_. After 30‐min fixation with methanol, the cells were subjected to 20‐min crystal violet (0.1%) staining and were observed under the inverted microscope. The number of transmembrane cells was counted in randomly selected five visual fields.

Invasion detection was performed. In brief, the extracellular matrix (ECM) gel was diluted using serum‐free culture medium at 1 : 9 to a final concentration of 1 mg·mL^−1^. The polycarbonate membrane in the 24‐well apical chamber was supplemented with 40 μL ECM gel and then further incubated at 37 °C with 5% CO_2_ for 5 h until the ECM gel was polymerized. A 70 μL portion of pure DMEM was then supplemented to the ECM gel, followed by further 0.5‐h incubation at 37 °C to hydrate the ECM gel. The starved osteosarcoma cells in serum for 24 h were resuspended with FBS‐free DMEM to a final concentration of 2.5 × 10^5^ cells·mL^−1^. Then, the hydrated basement membrane of the apical chamber and the basolateral chamber were added with 0.2 mL of cell suspension and 700 μL of precooled DMEM conjugated with 10% FBS, respectively. Then, 24‐h incubation of chambers was conducted at 37 °C with 5% CO_2_. After 30‐min methanol fixation, the cells were subjected to 20‐min crystal violet (0.1%) staining and observed under the inverted microscope. We randomly selected five visual fields to count the number of cells that had passed through the membranes.

### 2.10 Fluorescence *in situ* hybridization

Based on the protocols in the RiboTM lncRNA FISH Probe Mix (Red) Kit (Guangzhou RiboBio Co., Ltd., Guangzhou, Guangdong, China), fluorescence *in situ* hybridization (FISH) was operated to identify the subcellular location of PGM5‐AS1 expression in osteosarcoma cells. The osteosarcoma cells were positioned onto the slide in a 6‐well plate, followed by 1‐h culture till the cell confluence was about 80%. After fixation with 1 mL of 4% paraformaldehyde, the cells were manipulated with protease K (2 μg·mL^−1^), glycine, and acetylation reagent, and then incubated with 250 μL prehybridization. After the removal of the prehybridization, the cells were hybridized overnight with 250 μL hybridization solution supplemented with 300 ng·mL^−1^ probe. The fluorescence microscope (Olympus Optical, Tokyo, Japan) was applied for the observation of cells.

### 2.11 Fractionation of nuclear/cytoplasmic RNA

The osteosarcoma cells were resuspended with Hypotonic Buffer A [10 mm HEPES (pH = 7.5), 0.5 mm DTT, 10 mm KCl, 1.5 mm MgCl_2_] encompassing protease inhibitor and RNase inhibitor (N8080119; Thermo Fisher Scientific), followed by 10‐min incubation on ice and 10‐min centrifugation at 1000 ***g*** and 4 °C. The cytoplasm was separated by centrifuging the obtained supernatant at 15 000 ***g*** for 15 min. The precipitate was washed with hypotonic buffer and resuspended in Hypotonic Buffer B [10 mm HEPES (pH = 7.5), 10 mm KCl, 1.5 mm MgCl_2_, 0.5 mm DTT, 0.5% Nonidet P‐40] and radioimmunoprecipitation assay buffer [50 mm Tris/HCl (pH = 7.5), 1500 mm KCl, 1% Nonidet P‐40, 0.5% sodium deoxycholate, 0.1% sodium dodecyl sulfate, 1 mm ethylenediaminetetraacetic acid, pH = 8.0]. After 20‐min centrifugation of the precipitate at 15 000 ***g***, the supernatant containing the nuclear fraction was harvested.

### 2.12 RNA pull‐down assay

Following the guidelines of the Lipofectamine 2000 kits (11668019; Invitrogen, New York, Carlsbad, CA, USA), the cells were manipulated with 100 pmol Bio‐miR‐140‐5p or NC. After 48‐h transduction, the cells were resuspended in 0.7 mL lysis buffer [5 mm MgCl_2_, 100 mm KCl, 20 mm Tris (pH = 7.5), 0.3% NP‐40, 50 U of RNase OUT (Invitrogen), and complete protease suppressor cocktail (Roche Applied Science, Indianapolis, IN, USA)]. The cell lysate was separated by centrifuging cells at 10 000 ***g*** for 10 min. RNA pull‐down assay of miRNA was performed based on previously published methods (Lal *et al*., 2011; Wang *et al*., 2017). The expression of PGM5‐AS1 in Bio‐miR‐140‐5p or NC was assessed using RT‐qPCR.

### 2.13 RNA immunoprecipitation assay

The interaction among miR‐140‐5p, PGM5‐AS1, and FBN1 was identified with a RNA immunoprecipitation (RIP) assay kit (Millipore Inc., Bedford, MA, USA). Following treatment with lysis buffer (P0013B; Beyotime Biotechnology Co., Shanghai, China), the cells were subjected to 10‐min centrifugation at 35 068 ***g*** and 4 °C to harvest the supernatant. A large portion of cell extract was taken as the input, and the remainder was cultured with the antibody for coprecipitation as follows: After being resuspended in 100 μL RIP Wash Buffer, 50 μL magnetic beads were cultured with 5 μg antibody. The complex of bead and antibody was then resuspended using 900 μL RIP Wash Buffer, followed by overnight culture in 100 μL cell extraction at 4 °C. The beads–protein complex was obtained by placing the samples on the magnetic base. The antibodies used for the RIP assay were argonaute 2 (Ago2, ab32381, 1 : 50; Abcam Inc.), with IgG (1 : 100, ab109489; Abcam Inc.) used as the NC.

### 2.14 Dual‐luciferase reporter gene assay

The entire length of FBN1 3′UTR was amplified. The FBN1‐wild‐type (WT) vector was constructed by cloning the RT‐qPCR products into the polyclonal sites of the downstream gene of pmirGLO (Promega, Madison, WI, USA) using the endonuclease sites Spe I and Hind III. The target gene prediction databases TargetScan, mirDIP, miRDB, and miRmap were applied for prediction of the binding site between miR‐140‐5p and its target. FBN1‐mutant type (MUT) vector was constructed via site‐directed mutagenesis. Using Renilla luciferase expression vector pRL‐TK (TaKaRa Biotechnology Co. Ltd, Liaoning, China) as the internal control, the plasmids were cotransfected with luciferase reporter vectors into HEK‐293T cells, followed by measurement of luciferase activity in the Dual‐Luciferase Reporter Assay System (Promega).

### 2.15 Xenograft tumor in nude mice

Seventy‐two female BALB/c nude mice aged 3–4 weeks and weighing 14–18 g were housed at constant temperature (25–27 °C) with relative humidity (45–50%). Osteosarcoma cell line U2OS was not transfected as control, or transfected with sh‐NC, sh‐PGM5‐AS1 sh‐FBN1, mimic NC, or miR‐140‐5p mimic. After the construction of stably transfected U2OS cell, a mouse model of osteosarcoma was established by injecting 10 μL of cell suspension (2 × 10^6^ cells/well) into the right proximal tibia of the mice. The tumor volume was recorded every 6 days with calipers and calculated as follows: tumor volume = *a* × *b* ^2^/2 (*a*, the maximum diameter; *b*, the minimum diameter), and plotted as a graph. Thirty days after injection, the nude mice were euthanized, followed by isolation and weighing of their tumors. RT‐qPCR and western blot analysis were carried out to detect the expression levels of PGM5‐AS1, FBN1, miR‐140‐5p, and EMT‐related genes in tumor tissues. Organs were fixed with 2% formalin for 30 min at room temperature and then stained with X‐gal. The lung surface was stained using indigo, and the number of lung metastases was counted at 4× magnification with a Nikon Eclipse E600 microscope (Nikon, Tokyo, Japan).

### 2.16 Statistical analysis

The spss 21.0 software (IBM Corp., Armonk, NY, USA) was applied in data analysis. The measurement data were presented as mean ± standard deviation. The pair‐designed data between two groups conforming to normal distribution and homogeneity of variance were analyzed using a paired *t*‐test. One‐way analysis of variance (ANOVA), along with Tukey's *post hoc* test, was used for comparison of data among multiple groups. Repeated measurement ANOVA, together with Bonferroni's *post hoc* test, was conducted to analyze the data at different time points. The Kaplan–Meier method was adopted to construct the overall survival curve, and log‐rank was used for the analysis of the survival differences. The analysis of the enumeration data was performed using the chi‐square test. A *P* < 0.05 was required for results to be considered statistically significant.

## 3 Results

### 3.1 PGM5‐AS1 expression was elevated in osteosarcoma tissues and cells

Differentially expressed genes related to osteosarcoma were identified using the microarray dataset of GSE41445 from the GEO database, which revealed increased lncRNA PGM5‐AS1 expression in osteosarcoma samples through differential analysis of the gene expression in three normal samples and three osteosarcoma samples (Fig. 1A).

**Fig. 1:** The PGM5‐AS1 expression is elevated in osteosarcoma tissues and cells. (A) Expression of PGM5‐AS1 in normal samples and osteosarcoma samples retrieved from the microarray dataset GSE41445; the abscissa represents sample type, the ordinate represents the expression of PGM5‐AS1, and the number in the upper left represents the *P*‐value. (B) PGM5‐AS1 level in adjacent normal bone tissues and osteosarcoma tissues from 73 osteosarcoma patients measured by RT‐qPCR. (C, D) Expression location of PGM5‐AS1 in adjacent normal bone tissues and osteosarcoma tissues from 73 osteosarcoma patients identified using RNA *in situ* hybridization (*n* = 73, 400×; scale bar = 25 μm). (E) The relationship between PGM5‐AS1 expression and overall survival time of osteosarcoma patients analyzed using the Kaplan–Meier method. (F) Expression of PGM5‐AS1 in the normal cell line hFOB 1.19 and osteosarcoma cell lines (U2OS, SaOS‐2, MG63, HOS, and SJSA1), as determined by RT‐qPCR. *P < 0.05, *vs*. normal samples or hFOB 1.19 cell line. The measurement data were expressed as mean ± standard deviation. Data analysis in B was conducted by paired *t*‐test, data analysis in D by an unpaired *t*‐test, and data analysis in F by one‐way ANOVA, together with Tukey's *post hoc* test. Each reaction was run in triplicate.

To validate the microarray results, PGM5‐AS1 expression in osteosarcoma tissues collected from 73 osteosarcoma patients was determined using RT‐qPCR, which showed elevated expression of PGM5‐AS1 in osteosarcoma tissues compared to adjacent normal bone tissues (Fig. 1B). Besides, the situation of PGM5‐AS1 in osteosarcoma tissues and adjacent normal bone tissues was determined by RNA *in situ* hybridization, which exhibited that PGM5‐AS1 was located in the cytoplasm of osteosarcoma tissues with high expression (Fig. 1C,D). The osteosarcoma patients were assigned into patients with poor and high PGM5‐AS1 expression to assess this as a clinical indicator in osteosarcoma patients. PGM5‐AS1 expression was closely correlated to the tumor–node–metastasis stage, distant metastasis, tumor grade, and tumor size. However, PGM5‐AS1 expression does not correlate to the age and gender of the patients (Table 3). The Kaplan–Meier analysis showed that patients with poor PGM5‐AS1 level had longer survival time (log‐rank *P* < 0.05) (Fig. 1E). Additionally, we tested the PGM5‐AS1 expression in the normal cell line hFOB 1.19 and 5 osteosarcoma cell lines (U2OS, SaOS‐2, MG63, HOS, and SJSA1). The results indicated higher PGM5‐AS1 expression in osteosarcoma cell lines than in normal cell line hFOB 1.19 (*P* < 0.05) (Fig. 1F). The highest level of PGM5‐AS1 was observed in U2OS and HOS cells compared with SaOS‐2, MG63, and SJSA1 cells. Therefore, further assays were conducted on selected U2OS and HOS cells. In a word, PGM5‐AS1 was elevated in osteosarcoma tissues and cells.

**Table 3:** Relationship between PGM5‐AS1 expression and the clinical indicators of osteosarcoma patients. TNM, tumor–node–metastasis.

Clinicopathologic features	Cases (*n*)	PGM5‐AS1 expression		*P*‐value
		Low (*n* = 36)	High (*n* = 37)	
Age (years)				
≤ 20	33	18	15	0.484
> 20	40	18	22	
Gender				
Male	41	23	18	0.241
Female	32	13	19	
TNM stage				
I + II	48	30	18	0.003
III + IV	25	6	19	
Distant metastasis				
Yes	25	7	18	0.013
No	48	29	19	
Tumor grade				
Low	41	25	16	0.034
High	32	11	21	
Tumor size				
≤ 5cm	38	26	12	0.001
> 5cm	35	10	25	

### 3.2 Knocking down PGM5‐AS1 hinders osteosarcoma cell abilities of EMT, invasion, and migration

With the aspiration to reveal the mechanism by which PGM5‐AS1 affects EMT, invasion, and migration of osteosarcoma cells, we used shRNA to alter the level of PGM5‐AS1 in U2OS and HOS cells. According to RT‐qPCR, sh‐PGM5‐AS1‐1 treatment and sh‐PGM5‐AS1‐2 treatment reduce PGM5‐AS1 level in U2OS and HOS cells (Fig. 2A). As revealed by RT‐qPCR and western blot analysis, PGM5‐AS1 knockdown decreased the levels of N‐cadherin and Vimentin, while elevating the level of E‐cadherin in U2OS and HOS cells (Fig. 2B,C). Then, Transwell assay illustrated that decreasing PGM5‐AS1 reduced the invasion and migration abilities in U2OS and HOS cells (Fig. 2D,E). Thus, depleting the expression of PGM5‐AS1 dampens osteosarcoma cell EMT, invasion, and migration.

**Fig. 2:** Depleting PGM5‐AS1 attenuated osteosarcoma cell EMT, invasion, and migration. sh‐NC, sh‐PGM5‐AS1‐1, or sh‐PGM5‐AS1‐2 was delivered into U2OS and HOS cells. (A) Expression of PGM5‐AS1 in U2OS and HOS cells, as measured using RT‐qPCR. (B) Relative expression of EMT‐related genes in U2OS and HOS cells detected by RT‐qPCR. (C) Protein expression of EMT‐related genes in U2OS and HOS cells detected by western blot analysis. (D) Migration ability of U2OS and HOS cells detected by Transwell assay (200×; scale bar = 50 μm). (E) Invasion ability of U2OS and HOS cells detected by Transwell assay (200×; scale bar = 50 μm). *P < 0.05, *vs*. U2OS and HOS cells manipulated with sh‐NC. The measurement data were presented as mean ± standard deviation. One‐way ANOVA along with Tukey's *post hoc* test was conducted to analyze the data among multiple groups. The experiment was repeated three times.

### 3.3 The elevation of PGM5‐AS1 promotes osteosarcoma cell abilities of EMT, invasion, and migration

To elucidate better the role of PGM5‐AS1 osteosarcoma cells, PGM5‐AS1 was overexpressed in U2OS and HOS cells. RT‐qPCR results revealed that oe‐PGM5‐AS1 treatment markedly increased PGM5‐AS1 expression (Fig. 3A). Based on RT‐qPCR and western blot analysis, PGM5‐AS1 overexpression enhanced the levels of N‐cadherin and Vimentin, but diminished the level of E‐cadherin in U2OS and HOS cells (Fig. 3B,C). Transwell assay results indicated that oe‐PGM5‐AS1 treatment increased the abilities of invasion and migration in U2OS and HOS cells (Fig. 3D,E). Thus, elevation of PGM5‐AS1 promotes osteosarcoma cell EMT, invasion, and migration.

**Fig. 3:** PGM5‐AS1 upregulation exacerbated osteosarcoma cell EMT, invasion, and migration. oe‐NC or oe‐PGM5‐AS1 was delivered into U2OS and HOS cells. (A) Expression of PGM5‐AS1 in U2OS and HOS cells, as measured using RT‐qPCR. (B) Relative mRNA expression of EMT‐related genes in U2OS and HOS cells detected by RT‐qPCR. (C) Protein expression of EMT‐related genes in U2OS and HOS cells detected by western blot analysis. (D) Migration ability of U2OS and HOS cells detected by Transwell assay (200×; scale bar = 50 μm). (E) Invasion ability of U2OS and HOS cells detected by Transwell assay (200×; scale bar = 50 μm). *P < 0.05, *vs*. U2OS and HOS cells treated with sh‐NC. The measurement data were presented as mean ± standard deviation. One‐way ANOVA along with Tukey's *post hoc* test was conducted to analyze the data among multiple groups. The experiment was repeated three times.

### 3.4 PGM5‐AS1 binds to miR‐140‐5p

Having explored the role of PGM5‐AS1 in osteosarcoma, we turned to evaluate the relationship between PGM5‐AS1 and miR‐140‐5p. As shown by RNA *in situ* hybridization, PGM5‐AS1 expression was mostly found in the cytoplasm (Fig. 4A), which was further confirmed by FISH results (Fig. 4B) and fractionation of nuclear/cytoplasmic RNA (Fig. 4C). Moreover, the downstream miRNAs of PGM5‐AS1 were predicted using the RAID database, which yielded nine miRNAs. Among these, miR‐140‐5p presented with the most significantly differential expression in osteosarcoma (Fig. 4D). Thus, we supposed that PGM5‐AS1 might influence the expression of miR‐140‐5p to orchestrate osteosarcoma progression. Indeed, many studies have associated miR‐140‐5p with the biological processes of cancers (Gullu *et al*., 2015; Lan *et al*., 2015; Wang *et al*., 2016). Therefore, we carried out RT‐qPCR and western blot analysis to test miR‐140‐5p expression, which revealed poor miR‐140‐5p expression in osteosarcoma tissues *vs*. that in the adjacent normal bone tissues (Fig. 4E). RT‐qPCR (Fig. 4F) also demonstrated that, compared with hFOB 1.19 cells, miR‐140‐5p expression was significantly reduced in U2OS, SaOS‐2, MG63, HOS, and SJSA1 cells (*P* < 0.05). As indicated by RNA *in situ* hybridization, miR‐140‐5p expression was diminished in the cytoplasm of osteosarcoma tissues (Fig. 4G). Furthermore, RNA pull‐down assay (Fig. 4H) and RIP assay (Fig. 4I) manifested that PGM5‐AS1 could bind to miR‐140‐5p. Taken together, the results verified that PGM5‐AS1 could bind to miR‐140‐5p.

**Fig. 4:** PGM5‐AS1 binds to miR‐140‐5p in osteosarcoma. (A) The expression location of PGM5‐AS1 analyzed using RNA *in situ* hybridization. PGM5‐AS1 expression in the cytoplasm was shown above the 0 line, and PGM5‐AS1 expression in the nucleus was shown under the 0 line. (B) The location of PGM5‐AS1 expression in U2OS cells detected using FISH (200×; scale bar = 50 μm). (C) The location of PGM5‐AS1 expression in U2OS and HOS cells analyzed by fractionation of nuclear/cytoplasmic RNA. (D) Regulatory miRNA of PGM5‐AS1 predicted using the RAID database. (E) miR‐140‐5p level in osteosarcoma tissues and adjacent normal bone tissues from 73 osteosarcoma patients determined by RT‐qPCR. (F) The expression of miR‐140‐5p in human normal cell line hFOB 1.19 and five osteosarcoma cell lines U2OS, SaOS‐2, MG63, HOS, and SJSA1 detected by RT‐qPCR. *P < 0.05, *vs*. human normal cell line hFOB 1.19 cells. (G) Expression of miR‐140‐5p in osteosarcoma tissues from 73 osteosarcoma patients, as measured using RNA *in situ* hybridization (*n* = 73; 400×; scale bar = 25 μm). (H) The binding between miR‐140‐5p and PGM5‐AS1 detected by RNA pull‐down assay. (I) The binding between miR‐140‐5p and PGM5‐AS1 detected by RIP assay. *P < 0.05, *vs*. U2OS and HOS cells treated with sh‐NC, adjacent normal bone tissues, Bio‐NC, or IgG. The data were measurement data and expressed as mean ± standard deviation. Data in E were analyzed using *t*‐test. Unpaired *t*‐test was used to analyze the data between the two groups, and one‐way ANOVA together with Tukey's *post hoc* test was applied in data analysis among multiple groups. The experiment was repeated three times.

### 3.5 Depleted PGM5‐AS1 expression contributes to repressed osteosarcoma progression by competitively binding to miR‐140‐5p

In order to identify the promising influence of PGM5‐AS1 in the progression of osteosarcoma, we first carried out RT‐qPCR to measure the levels of PGM5‐AS1 and miR‐140‐5p in U2OS and HOS cells (Fig. 5A). The expression patterns of genes associated with EMT including E‐cadherin, N‐cadherin, and Vimentin were detected by performing RT‐qPCR and western blot analysis, which showed that knocking down miR‐140‐5p reduced E‐cadherin expression, but elevated N‐cadherin and Vimentin expression (Fig. 5B,C). Next, Transwell assay showed promotion in migration and invasion in osteosarcoma cells (Fig. 5D,E). PGM5‐AS1 reduction resulted in upregulated E‐cadherin expression, downregulated expression of N‐cadherin and Vimentin (Fig. 5B,C), and attenuated migration and invasion in osteosarcoma cells (Fig. 5D,E). Cotreatment of silenced PGM5‐AS1 and reduced miR‐140‐5p rescued the suppressive role in osteosarcoma cell invasion and migration. Therefore, knockdown of PGM5‐AS1 upregulates miR‐140‐5p, thus inhibiting osteosarcoma progression.

**Fig. 5:** Silencing of PGM5‐AS1 upregulates miR‐140‐5p to suppress the progression of osteosarcoma. The si‐PGM5‐AS1‐1 and miR‐140‐5p inhibitor, as well as the corresponding NC, were delivered into the U2OS and HOS cells. (A) Expression of PGM5‐AS1, miR‐140‐5p, and FBN1 in U2OS and HOS cells detected by RT‐qPCR. (B) RT‐qPCR results of EMT‐related gene expression (E‐cadherin, N‐cadherin, and Vimentin) in U2OS and HOS cells. (C) Western blot analysis of EMT‐related gene protein expression (E‐cadherin, N‐cadherin, and Vimentin) in U2OS and HOS cells. (D) Migration ability of U2OS and HOS cells assessed by Transwell assay (200×; scale bar = 50 μm). (E) Invasion ability of U2OS and HOS cells assessed by Transwell assay (200×; scale bar = 50 μm). *P < 0.05, *vs*. U2OS and HOS cells treated with both si‐NC and inhibitor NC; ^#^ *P* < 0.05, *vs*. U2OS and HOS cells treated with both si‐PGM5‐AS1‐1 and inhibitor NC. The data were measurement data and expressed as mean ± standard deviation. One‐way ANOVA as well as Tukey's *post hoc* test was used for data analysis among multiple groups. The experiment was repeated three times.

### 3.6 FBN1 is the target of miR‐140‐5p

The target of miR‐140‐5p and their interaction were predicted and verified using dual‐luciferase reporter gene assay, RNA pull‐down assay, and RIP assay. The predicted results and the upregulated genes retrieved from the microarray dataset GSE41445 showed three genes in the intersection, which might be targeted and regulated by miR‐140‐5p (Fig. 6A). From RT‐qPCR results, FBN1 expression was the most significantly differential in osteosarcoma (Fig. 6B). RT‐qPCR exhibited that osteosarcoma tissues indeed had elevated expression of FBN1 *vs*. the adjacent normal bone tissues (Fig. 6C). RT‐qPCR results also depicted that, compared with hFOB 1.19 cells, FBN1 mRNA expression was markedly elevated in U2OS, SaOS‐2, MG63, HOS, and SJSA1 cells (*P* < 0.05; Fig. 6D). U2OS cells were then transfected with plasmids containing miR‐140‐5p mimic or miR‐140‐5p inhibitor, and the expression of FBN1 was measured. Results revealed that enforced expression of miR‐140‐5p led to FBN1 depletion, which was opposite to reduced expression of miR‐140‐5p (Fig. 6E,F). Knocking down PGM5‐AS1 reduced the FBN1 content, which was annulled by miR‐140‐5p silencing. As determined by dual‐luciferase reporter gene assay, overexpressing miR‐140‐5p decreased but suppressing miR‐140‐5p potentiated the luciferase activity of FBN1‐WT without affecting luciferase activity of FBN1‐MUT (Fig. 6G). Repressing both miR‐140‐5p and PGM5‐AS1 rescued the downregulatory effect of miR‐140‐5p on luciferase activity (Fig. 6H). Furthermore, RIP assay revealed that miR‐140‐5p could bind to FBN1 (Fig. 6I) and PGM5‐AS1 silencing enhanced the binding of miR‐140‐5p to FBN1 (Fig. 6J,K). These results provide evidence that miR‐140‐5p specifically targets FBN1.

**Fig. 6:** miR‐140‐5p negatively modulates FBN1 expression. Mimic or inhibitor or shRNA was used to interfere with the levels of miR‐140‐5p and PGM5‐AS1 in U2OS cells. (A) Prediction results of the gene targeted by miR‐140‐5p. The ovals represent the predicted results and the upregulated genes in the microarray dataset GSE41445. The overlapping section refers to the intersection of the five ovals. (B) Expression of MMP, FBN1, and KLF9 in U2OS cells with altered PGM5‐AS1 expression detected by RT‐qPCR. (C) FBN1 level in osteosarcoma tissues and adjacent normal bone tissues from 73 osteosarcoma patients tested using RT‐qPCR. (D) The mRNA expression of FBN1 in human normal cell line hFOB 1.19 and five osteosarcoma cell lines U2OS, SaOS‐2, MG63, HOS, and SJSA1. *P < 0.05, *vs*. human normal cell line hFOB 1.19 cells. (E) Relative expression of FBN1 in U2OS cells with altered miR‐140‐5p expression detected by RT‐qPCR. (F) Protein expression of FBN1 in U2OS cells with altered miR‐140‐5p expression detected by western blot analysis. (G) The binding of miR‐140‐5p and FBN1 confirmed by dual‐luciferase reporter gene assay. (H, I) Luciferase activity of FBN1 measured by dual‐luciferase reporter gene assay. (J) Interaction between miR‐140‐5p and FBN1 in U2OS cells as detected by RIP assay. (K) Interaction between miR‐140‐5p and FBN1 in U2OS cells with altered PGM5‐AS1 expression as measured using RIP assay. *P < 0.05, *vs*. U2OS cells treated with sh‐NC, adjacent normal bone tissues, IgG treatment, or U2OS cells treated with both sh‐NC and inhibitor NC; ^#^ *P* < 0.05, *vs*. U2OS cells administered with inhibitor NC or AGO2 enrichment in sh‐NC. The measurement data were expressed as mean ± standard deviation. The data in C were analyzed using the paired *t*‐test. Unpaired *t*‐test was employed for data analysis between two groups and one‐way ANOVA, as well as Tukey's *post hoc* test for comparison of data among multiple groups. The experiment was repeated three times.

### 3.7 Restored expression of miR‐140‐5p reduces FBN1 to dampen processes of osteosarcoma

To elucidate better the effect of the miR‐140‐5p‐FBN1 axis on osteosarcoma progression, we adopted RT‐qPCR (Fig. 7A) and western blot analysis (Fig. 7B) to test the levels of FBN1 and genes linked to EMT, like E‐cadherin, N‐cadherin, and Vimentin (Fig. 7C,D). We also used the Transwell assay (Fig. 7E,F) to examine invasion and migration in osteosarcoma cells. Results revealed that depleting FBN1 diminished FBN1, N‐cadherin, and Vimentin expression, but enhanced E‐cadherin expression, and attenuated the invasion and migration in osteosarcoma cells. Conversely, knockdown of miR‐140‐5p resulted in elevation in FBN1, N‐cadherin, and Vimentin expression, reduction in E‐cadherin, and promotion in invasion and migration abilities of osteosarcoma cells. Depletion of FBN1 as well as depletion miR‐140‐5p rescued the suppressive role of FBN1 in invasion and migration of osteosarcoma cells. In summary, the upregulation of miR‐140‐5p decreased FBN1 expression to inhibit the progression of osteosarcoma.

**Fig. 7:** miR‐140‐5p upregulation hindered the expression of FBN1 to dampen osteosarcoma progression. The expression of miR‐140‐5p in U2OS and HOS cells was altered with inhibitor, and the expression of FBN1 was altered with shRNA. (A) Relative expression of FBN1 in U2OS and HOS cells measured using RT‐qPCR. (B) Protein expression of FBN1 in U2OS and HOS cells detected by western blot analysis. (C) Expression of genes related to EMT including E‐cadherin, N‐cadherin, and Vimentin in U2OS and HOS cells measured using RT‐qPCR. (D) Protein levels of EMT‐related genes (E‐cadherin, N‐cadherin, and Vimentin) in U2OS and HOS cells detected by western blot analysis. (E) Migration ability of U2OS and HOS cells measured by Transwell assay (200×; scale bar = 50 μm). (F) Invasion ability of U2OS and HOS cells measured by Transwell assay (200×; scale bar = 50 μm). *P < 0.05, *vs*. U2OS cells treated with combined sh‐NC and inhibitor NC; ^#^ *P* < 0.05, *vs*. U2OS cells treated with combined sh‐FBN1 and sh‐NC. The data were measurement data and expressed as mean ± standard deviation. Data among multiple groups were analyzed using one‐way ANOVA, followed by Tukey's *post hoc* test. The experiment was repeated three times.

### 3.8 PGM5‐AS1 silencing, FBN1 silencing, or miR‐140‐5p overexpression inhibits tumorigenesis of osteosarcoma cells *in vivo*

The role of PGM5‐AS1 in osteosarcoma *in vivo* was also assessed. Based on the tumor volume and weight, it was found that PGM5‐AS1 silencing, FBN1 silencing, or miR‐140‐5p overexpression inhibited tumorigenesis of osteosarcoma cells (Fig. 8A). RT‐qPCR revealed that si‐PGM5‐AS1 treatment reduced the levels of PGM5‐AS1 and FBN1 and elevated the expression of miR‐140‐5p. Treatment with miR‐140‐5p mimic resulted in elevated miR‐140‐5p expression and declined FBN1 levels, while the expression of PGM5‐AS1 remained unchanged. Silencing of FBN1 diminished FBN1 expression, while the expression of PGM5‐AS1 and miR‐140‐5p remained unchanged (Fig. 8B). Moreover, RT‐qPCR and western blot analysis showed that PGM5‐AS1 silencing, FBN1 silencing, or miR‐140‐5p overexpression contributed to marked elevation of E‐cadherin content and reduction of the contents of N‐cadherin and Vimentin (Fig. 8C,D). Moreover, we counted the number of lung metastases in nude mice, and results displayed that silencing PGM5‐AS1 or FBN1, or overexpressing miR‐140‐5p reduced the number of lung metastases (Fig. 8E). Thus, PGM5‐AS1 silencing results in inhibited tumorigenesis in osteosarcoma cells *in vivo* via miR‐140‐5p‐targeted FBN1.

**Fig. 8:** Tumorigenesis of osteosarcoma cells *in vivo* is suppressed by the downregulation of PGM5‐AS1 or FBN1 or overexpression of miR‐140‐5p. (A) Tumor volume and tumor weight of the nude mice. (B) Expression of PGM5‐AS1, FBN1, and miR‐140‐5p in developed tumors detected by RT‐qPCR. (C) Expression patters of genes related to EMT including E‐cadherin, N‐cadherin, and Vimentin tested using RT‐qPCR. (D) Protein expression of EMT‐related genes (E‐cadherin, N‐cadherin, and Vimentin) as measured by western blot analysis. (E) Micrographs (left) and number (right) of tumor lung metastases of nude mice (400×; scale bar = 25 μm). *P < 0.05, *vs*. the nude mice injected with sh‐NC‐treated U2OS cells. The data were measurement data and expressed as mean ± standard deviation. Unpaired *t*‐test was performed to compare the data between two groups, and repeated measurement ANOVA along with Bonferroni's *post hoc* test was conducted for analysis of data at different time points. *n* = 12.

## 4 Discussion

Osteosarcoma possesses a poor survival rate despite recent improvements in its diagnosis and management (Geller and Gorlick, 2010). Hence, we are motivated to find out effective biological markers that could improve osteosarcoma management. Recently, it is extensively accepted that a variety of lncRNAs and miRNAs critically influence the progression of osteosarcoma (Wang *et al*., 2018a, 2018b,2018a, 2018b). However, there has been no study elucidating the underlying mechanism of PGM5‐AS1 in osteosarcoma. Thus, we performed the present study to reveal the specific mechanisms of PGM5‐AS1 in the network of lncRNA‐miRNA‐mRNA in osteosarcoma. Intriguingly, our results proved that silencing PGM5‐AS1 elevates the expression of miR‐140‐5p, which in turn reduces the FBN1 level, thus attenuating invasion and EMT of osteosarcoma.

Initially, we found elevated expression of PGM5‐AS1 and FBN1 but reduced expression of miR‐140‐5p in osteosarcoma tissues and cells. Diverse lncRNAs have been widely elucidated to be upregulated in osteosarcoma. For instance, levels of both HULC and UCA1 were elevated in osteosarcoma cells and tissues, and the upregulation of these two lncRNAs was correlated with metastasis and clinical stage of osteosarcoma (Li *et al*., 2016; Sun *et al*., 2015). Consistent with that finding, the PGM5‐AS1 is an upregulated gene in anaplastic glioma (Wang *et al*., 2018a, 2018b,2018a, 2018b). Also, upregulation of PGM5‐AS1 also occurs in colorectal cancer and is linked to poor survival rate of colorectal cancer patients (Zhu *et al*., 2017a, 2017b,2017a, 2017b). Besides, osteosarcoma cells display increased expression of FBN1 (Han *et al*., 2014; Summers *et al*., 2009). Likewise, the levels of FBN1 were increased in the tissues and cells in gastric cancer, and its reduction attenuated the progression of gastric cancer (Yang *et al*., 2017). Moreover, Meng *et al*. (2017) found that the miR‐140‐5p level was linked to chemosensitivity in osteosarcoma, whereby downregulated miR‐140‐5p expression occurred following chemotherapy.

Another key finding in our study is that PGM5‐AS1 was confirmed to bind competitively to miR‐140‐5p, thus increasing FBN1 expression. In agreement with the present results, an earlier study showed that lncRNA ODRUL upregulated MMP2 by directly downregulating miR‐3182 to further induce the progression of osteosarcoma (Zhu *et al*., 2017a, 2017b,2017a, 2017b). Also, the depletion of SNHG12 upregulated miR‐195‐5p to downregulate Notch2, thus suppressing the progression of osteosarcoma (Zhou *et al*., 2018). Moreover, Ma *et al*. revealed that FBN1 was a target gene of miR‐486‐5p, whereby the elevated expression of miR‐486‐5p could target FBN1 to suppress the development of papillary thyroid carcinoma (Ma *et al*., 2016). Also, miR‐140‐5p negatively regulated IP3k2 to suppress autophagy in osteosarcoma after chemotherapy (Wei *et al*., 2016).

Furthermore, our results revealed that depleting the expression of PGM5‐AS1 or FBN1, or enforcing the expression of miR‐140‐5p repressed osteosarcoma cell migration, invasion, and EMT of *in vitro* and attenuated tumorigenesis *in vivo*. In accordance with our results, a previous study showed that reduced DANCR downregulated ALX to inhibit cell proliferation, invasion, and migration *in vitro*, as well as suppressing osteosarcoma tumor growth *in vivo* by specifically upregulating miR‐33a‐5p (Jiang *et al*., 2017). Similarly, the depletion of lncRNA prostate cancer‐associated transcript 1 has led to the repressed cell invasion, migration, proliferation, and EMT of osteosarcoma cells (Zhang *et al*., 2018a, 2018b,2018a, 2018b). Also, ovarian cancer cell migration and invasion were revealed to be attenuated following FBN1 silencing (Wang *et al*., 2015). Consistent with those results, upregulation of miR‐140 negatively mediated the expression of histone deacetylase 4, leading to inhibited osteosarcoma cell proliferation and invasion *in vitro* and slowed tumor growth *in vivo*, which together highlighted overexpressed miR‐140 as a tumor inhibitor in osteosarcoma (Xiao *et al*., 2017). Likewise, miR‐140 was indicated to be a suppressor in osteosarcoma owing to its role in repressing proliferation, migration, and tumor aggressiveness (Gu *et al*., 2016). Furthermore, Zhang *et al*. (2018a, 2018b,2018a, 2018b) confirmed that the depleting the expression of small nucleolar RNA host gene 16 led to increased miR‐140‐5p levels, thus downregulating ZEB1 and thereby dampening esophageal squamous cell carcinoma cell proliferation, migration, and EMT.

## 5 Conclusion

Taken together, our findings provide new evidence demonstrating that the depleted PGM5‐AS1 competitively binds to miR‐140‐5p, resulting in the decreased expression of FBN1 and suppressed osteosarcoma progression (Fig. 9). Our novel results indicate this pathway as a potential biological marker better to manage osteosarcoma and also lay a theoretical foundation for elucidating the specific mechanisms of various lncRNAs in osteosarcoma. However, more in‐depth investigations of the PGM5‐AS1/miR‐140‐5p/FBN1 axis are required before translation to clinical practice. Moreover, the downstream pathways of the PGM5‐AS1 in osteosarcoma should be identified in future studies.

**Fig. 9:** Modulatory role of PGM5‐AS1 in the cellular processes of osteosarcoma by interacting with miR‐140‐5p and FBN1. Knocking down the expression of PGM5‐AS1 specifically binds to miR‐140‐5p to silence the level of FBN1 and thereby attenuate EMT, invasion, and migration of osteosarcoma *in vitro* as well as tumorigenesis *in vivo*.

## Conflict of interest

The authors declare no conflict of interest.

## Author contributions

WL and PL designed the study. HG, XW, and MY collated the data, carried out data analyses, and produced the initial draft of the manuscript. WL, PL, and MY contributed to drafting the manuscript. All authors have read and approved the final submitted manuscript.

## Data Availability

The data that support the findings of this study are available in this article.
